RETRACTED

# Novel Single Nucleotide Polymorphisms in Interleukin 6 Affect Tacrolimus Metabolism in Liver Transplant Patients

**DOI:** 10.1371/journal.pone.0073405

**Published:** 2013-08-26

**Authors:** Dawei Chen, Junwei Fan, Feng Guo, Shengying Qin, Zhaowen Wang, Zhihai Peng

**Affiliations:** 1 Department of General Surgery, Shanghai First People's Hospital, School of Medicine, Shanghai Jiao Tong University, Shanghai, China; 2 Key Laboratory for the Genetics of Developmental and Neuropsychiatric Disorders, Bio-X Institutes, Ministry of Education, Shanghai Jiao Tong University; Shanghai Genomepilot Institutes for Genomics and Human Health, Shanghai, China; The University of Hong Kong, Hong Kong

## Abstract

**Background:**

Tacrolimus is the first-line immunosuppressant after organ transplantation. It is mainly metabolized by cytochrome P450, family 3, subfamily A (CYP3A) enzymes, but there are large individual differences in metabolism. Interleukin 6 (IL6) has been shown to cause a pan-suppression of mRNA levels of ten major CYP enzymes in human hepatocyte cultures. IL6 has been shown to provide hepatoprotection in various models of liver injury. Rs1800796 is a locus in the IL6 gene promoter region which regulates cytokine production. We speculated that IL6 rs1800796 polymorphisms may lead to individual differences in tacrolimus metabolism by affecting CYP3A enzymes levels and liver function after liver transplantation.

**Methodology/Principal Findings:**

Ninety-six liver transplant patients receiving tacrolimus were enrolled in the study. Two single nucleotide polymorphisms (SNP), CYP3A5 rs776746 and IL6 rs1800796, were genotyped in both donors and recipients. The effects of SNPs on tacrolimus concentration/dose (C/D ratio) at four weeks after transplantation were studied, as well as the effects of donor IL6 rs1800796 polymorphisms on liver function. Both donor and recipient CYP3A5 rs776746 allele A showed association with lower C/D ratios, while donor IL6 rs1800796 allele G showed an association with higher C/D ratios. Donor CYP3A5 rs776746 allele A, IL6 rs1800796 allele C, and recipient CYP3A5 rs776746 allele A were associated with fast tacrolimus metabolism. With increasing numbers of these alleles, patients were found to have increasingly lower tacrolimus C/D ratios at time points after transplantation. Donor IL6 rs1800796 allele G carriers showed an association with higher glutamic-pyruvic transaminase (GPT) levels.

**Conclusions:**

Combined analysis of donor CYP3A5 rs776746, IL6 rs1800796, and recipient CYP3A5 rs776746 polymorphisms may distinguish tacrolimus metabolism better than CYP3A5 rs776746 alone. IL6 may lead to individual differences in tacrolimus metabolism mainly by affecting liver function.

RETRACTED

## Introduction

Tacrolimus is the first-line immunosuppressant after organ transplantation, reducing rejection and improving graft and recipient survival. However, it is also characterized by a narrow therapeutic window, and large individual differences in metabolism [1], [2]. Indeed, after administration of “standard” doses, some patients show no therapeutic effects or serious side effects. Individualization of medical treatment could result in great improvement in therapeutic efficacy, and reduction of side effects, as well as reduction of the cost of treatment [3], [4]. At present, it is difficult to institute individualized medicine in the early postoperative period. Genetic factors such as polymorphisms can be closely related to drug metabolism. There is growing interest in the field of pharmacogenomics which focuses on the relationship between host genetics and drug metabolism [5]. Large clinical studies have shown that genetic factors can guide individualized medication of warfarin and clopidogrel [6], [7]. Pharmacogenomics research on tacrolimus could contribute to individualized medication in the early postoperative period of liver transplantation.

CYP3A enzymes, which are mainly expressed in liver and intestine, are the major metabolic enzymes of tacrolimus [8], [9]. The rs776746 polymorphisms in intron 3 of CYP3A5 have been correlated with altered gene expression due to a splicing defect. These CYP3A5 rs776746 GG genotype carriers are associated with slow tacrolimus metabolism [10], [11]. However, the effect by CYP3A5 rs776746 still does not completely explain individual differences in tacrolimus metabolism [12], [13].

IL6 has been demonstrated to cause a pan-suppression of mRNA of ten major CYP enzymes in human hepatocyte cultures [14]. IL6 could promote hepatic survival by stimulating liver regeneration and providing hepatoprotection in various models of liver injury [15], so it may be relevant to liver function after liver transplantation. The rs1800796 locus, which is in the IL6 gene promoter region, could regulate cytokine production and has been proved to be a functional SNP [16], [17].

The aim of the study was to investigate the relationship between tacrolimus metabolism and IL6 rs1800796 in a large liver transplant cohort to evaluate the possibility of individualizing tacrolimus treatment in the early postoperative period of liver transplantation.

## Materials and Methods

### Patients

A total of 96 patients (16 female and 80 male) who underwent liver transplantation at Shanghai Jiao Tong University Affiliated First People's Hospital between July 2007 and February 2011 were enrolled in this study. One patient was excluded from further analysis because the genotyping failed. The patients were all Han Chinese. The average age of the patients was 47.8±8.3 years, and the average weight was 63.0±10.4 kg. All of the patients received tacrolimus-based immunosuppressive regimens. Tacrolimus (Prograf, Astellas Pharma, Japan) was administered orally twice daily at an initial dose of 0.06 mg/kg/d. The dose of tacrolimus was adjusted according to the target blood concentration of 7 to10 ng/ml during the first month after transplantation.

RETRACTED

### Ethics Statement

This research was approved by the Ethics Committee of Shanghai Jiao Tong University, and informed written consent was obtained according to the Declaration of Helsinki and its amendments.

### Data Collection

Blood samples were collected half an hour before tacrolimus was administered, and trough concentrations (ng/ml) were then detected by PRO-Trac™ II Tacrolimus ELISA kit (Diasorin, USA) with microparticle enzyme immunoassay (ELx800NB analyzer, BioTek, USA). C/D ratio was calculated with trough concentration and weight standardized 24-hour tacrolimus dose (mg/kg/d). We calculated C/D ratios at four weeks after transplantation, and we used the median of C/D ratios at weeks 1 to 4 to measure weekly changes in tacrolimus metabolism. We also used the median of glutamic-pyruvic transaminase levels (U/L) at weeks 1 to 4 after transplantation to measure weekly liver function.

### Extracting genomic DNA and genotyping

Using an AllPrep DNA/RNA Mini Kit (Qiagen, Germany) according to the manufacturer’s instructions, genomic DNA was isolated from both donor and recipient liver tissue, where were previously stored at −80°C. Genotyping of SNPs was conducted by the Sequenom MassARRAY SNP genotyping platform (Sequenom, USA) [18]. The protocols included DNA and primer preparation, PCR amplification, SAP treatment, primer extension, resin cleanup, spotting primer extension products on SpectroCHIP, and detection primer extension products by mass spectrometer.

### Statistical Analysis

Hardy-Weinberg equilibrium and allele frequency were analyzed using PLINK v1.07 (http://pngu.mgh.harvard.edu/purcell/plink/). Quantitative data between two groups were compared using Mann-Whitney *U* tests, and among several groups by Kruskal-Wallis. Non-parametric tests were performed in SPSS v17.0 (SPSS, USA). Two-sided tests were used in all analysis, and *P*<0.05 was considered statistically significant.

## Results

### Gene polymorphisms

For CYP3A5, rs776746 allele A (28.4%) was found to be the minor allele, while allele G (71.6%) was the major allele. For IL6, rs1800796 allele G (30.3%) was found to be the minor allele, while allele C (69.7%) was the major allele. Both SNP frequencies were in accordance with Hardy-Weinberg equilibrium (*P*>0.05). There were no differences in allele frequencies of the two SNPs between donors and recipients. Genotype frequencies of the two SNPs are shown in Table 1.

RETRACTED

**Table 1:** Genotype frequencies of CYP3A5 rs776746 and IL6 rs1800796.

	Genotypes		Frequency of donors		Frequency of recipients	
SNPs	Ref^a^	Mut^b^	Ref	Mut	Ref	Mut
rs776746	GG	GA+AA	46(0.484)	49(0.516)	50(0.526)	45(0.474)
rs1800796	CC	CG+GG	41(0.432)	54(0.568)	49(0.516)	46(0.484)

a “Ref” is for referenced genotype, which is constituted of major allele and major allele. ^b^“Mut” is for mutated genotypes, which are constituted of major allele and minor allele or minor allele and minor allele.

### Associations between CYP3A5 rs776746, IL6 rs1800796 polymorphisms and tacrolimus C/D ratios

The effects of donor CYP3A5 rs776746 and IL6 rs1800796 polymorphisms on tacrolimus C/D ratios at four weeks after transplantation are shown in Table 2. Tacrolimus C/D ratios of donor CYP3A5 rs776746 allele A carriers at weeks 1, 3, and 4 were 199.0, 88.7, and 85.6, respectively, while C/D ratios of non-carriers were 295.1, 121.2, and 148.8, respectively. These differences between donor CYP3A5 rs776746 allele A carriers and non-carriers were significant (*P* = 0.006, 0.028, 0.001, respectively). Tacrolimus C/D ratios of donor IL6 rs1800796 allele G carriers at weeks 2 and 3 were 132.3 and 127.4, respectively, while C/D ratios of non-carriers were 105.2 and 97.4, respectively, and the differences were significant (*P* = 0.032, 0.021, respectively). Thus, donor CYP3A5 rs776746 allele A and IL6 rs1800796 allele C are associated with fast tacrolimus metabolism.

**Table 2:** The effects of donor CYP3A5 rs776746 and IL6 rs1800796 polymorphisms on tacrolimus C/D ratios.

			Week 1		Week 2		Week 3		Week 4	
SNPs	Genotypes	N	C/D ratio	*P*	C/D ratio	*P*	C/D ratio	*P*	C/D ratio	*P*
rs776746	GG	46	295.1±413.2	0.006	130.8±130.9	0.085	121.2±81.1	0.028	148.8±126.9	0.001
	GA+AA	49	199.0±209.8		102.8±101.1		88.7±102.5		85.6±75.5	
rs1800796	CC	41	221.2±275.0	0.314	105.2±91.1	0.032	97.4±76.1	0.021	95.1±83.7	0.113
	CG+GG	54	240.9±318.7		132.3±119.0		127.4±125.3		133.2±119.3	

The effects of recipient CYP3A5 rs776746 and IL6 rs1800796 polymorphisms on tacrolimus C/D ratios at four weeks after transplantation are shown in Table 3. Tacrolimus C/D ratios of recipient CYP3A5 rs776746 allele A carriers at weeks 1, 2, 3, and 4 were 179.0, 100.6, 97.0, and 90.2, respectively, while C/D ratios of non-carriers were 290.5, 133.2, 123.7, and 136.5, respectively, and the differences were significant (*P* = 0.003, 0.018, 0.030, 0.017, respectively). There was no significant difference in tacrolimus C/D ratio between recipient IL6 rs1800796 allele G carriers and non-carriers. Thus, recipient CYP3A5 rs776746 allele A is also associated with fast tacrolimus metabolism.

RETRACTED

**Table 3:** The effects of recipient CYP3A5 rs776746 and IL6 rs1800796 polymorphisms on tacrolimus C/D ratios.

			Week 1		Week 2		Week 3		Week 4	
SNPs	Genotypes	N	C/D ratio	*P*	C/D ratio	*P*	C/D ratio	*P*	C/D ratio	*P*
rs776746	GG	50	290.5±283.4	0.003	133.2±107.8	0.018	123.7±113.0	0.030	136.5±114.0	0.017
	GA+AA	45	179.0±237.5		100.6±105.7		97.0±82.9		90.2±83.0	
rs1800796	CC	49	282.6±338.3	0.217	133.3±142.5	0.344	110.6±110.8	0.604	133.1±144.4	0.135
	CG+GG	46	208.7±260.8		115.0±64.7		109.6±90.4		95.7±94.0	

### Associations between combined polymorphisms and tacrolimus C/D ratios

Donor CYP3A5 rs776746 allele A, IL6 rs1800796 allele C, and recipient CYP3A5 rs776746 allele A were shown to be associated with fast tacrolimus metabolism as stated above. Therefore, these three alleles were further investigated in a combination analysis. The associations between the number of alleles associated with fast metabolism and tacrolimus C/D ratios are shown in Table 4. With increasing numbers of alleles associated with fast metabolism, patients were found to have increasingly lower tacrolimus C/D ratios at all time points through the four weeks (*P* = 0.001, 0.001, <0.001, <0.001, respectively).

**Table 4:** Combined analysis of donor CYP3A5 rs776746 allele A, IL6 rs1800796 allele C, and recipient CYP3A5 rs776746 allele A on tacrolimus C/D ratios.

		Week 1		Week 2		Week 3		Week 4	
Num^a^	N	C/D ratio	*P*	C/D ratio	*P*	C/D ratio	*P*	C/D ratio	*P*
≤1	19	460.0±420.9	0.001	186.5±121.7	0.001	177.7±140.8	<0.001	172.5±177.6	<0.001
2−3	61	242.4±261.0		117.2±96.4		109.6±88.7		107.2±81.1	
≥4	15	91.8±167.9		59.0±93.6		67.7±49.0		73.4±47.9	

a “Num” indicates the number of alleles associated with fast metabolism patients carrying.

### Associations between donor IL6 rs1800796 polymorphisms and GPT

The effects of donor IL6 rs1800796 polymorphisms on GPT at four weeks after transplantation were studied. GPT of donor IL6 rs1800796 allele G carriers at weeks 1, 2, 3, and 4 were 167.0, 45.5, 30.0, and 34.5, respectively, while GPT of non-carriers were 142.5, 29.0, 20.0, and 20.0, respectively. The differences between donor IL6 rs1800796 allele G carriers and non-carriers at weeks 2, 3, and 4 were significant (*P* = 0.004, 0.002, 0.006, respectively), but not at week 1 (*P* = 0.141).

## Discussion

The CYP3A enzymes including three functional enzymes as CYP3A4, CYP3A5, and CYP3A7 are responsible for the oxidative metabolism of over 50% of the drugs in widespread use [19]. CYP3A4 is responsible for most CYP3A-mediated drug metabolism [20]. There have been previous studies on the associations between CYP3A4 gene polymorphisms and tacrolimus metabolism [21]–[23], but there are no definitive conclusions comparing with CYP3A5 rs776746. CYP3A7 is predominantly expressed in fetal liver and may have little role in adults [19]. CYP3A5 is the major metabolic enzyme for tacrolimus. CYP3A5 rs776746 allele A non-carriers produce truncated, nonfunctional CYP3A5 enzyme because of a splicing defect, so these patients metabolize tacrolimus slower than carriers [10], [11]. This dose-modifying effect in Eastern Asian populations is higher than in Caucasian populations [10]. In a study by Birdwell et al, eight SNPs in the CYP3A4 gene and one in the CYP3A7 gene were found to be associated with tacrolimus metabolism, but these SNPs were in linkage disequilibrium with CYP3A5 rs776746 [12]. CYP3A5 enzyme is expressed both in liver and intestine [24], so tacrolimus metabolism is associated with both donor and recipient CYP3A5 gene polymorphisms in liver transplant patients [10], [11]. Our study has verified that both donor and recipient CY3A5 rs776746 were associated with tacrolimus metabolism in a transplant population.

RETRACTED

It has been shown previously that CYP3A5 rs776746 could predict tacrolimus metabolism to a certain extent, but could not completely explain the individual differences [12], [13]. Presently, about two hundred cytokines produced by many cell types have been found, and they usually act by autocrine and paracrine mechanisms [25]. In recent years, more attention has been paid to relationships between cytokines and tacrolimus metabolism. There have been reports that donor and recipient IL10 gene polymorphisms were associated with tacrolimus metabolism and IL18 was thought to reduce tacrolimus C/D ratios through up regulation of P-glycoprotein [8], [26], [27]. Our study is the first to demonstrate that donor IL6 rs1800796 polymorphisms are associated with tacrolimus metabolism.

Previous studies have shown that cytokines affect pharmacokinetic and pharmacodynamic behaviors of drugs [25], [28]. IL6 has been shown to suppress mRNA of CYP3A5 in human hepatocyte cultures [14]. Cytokines also play a central role in immunologic events that occur after transplantation [29]. The liver often undergoes ischemia/reperfusion and immune injury during the transplantation and postoperative time. In this regard, IL6 activates the STAT3 signaling pathway through the gp130-IL6R complex on hepatocytes, and this process promotes liver regeneration, the acute-phase response, and hepatoprotection against Fas and toxic damage in liver [15]. Cytokine production may differ among different people due to gene polymorphisms [30], [31]. The rs1800796 locus in IL6 promoter, which can regulate its production, was shown to be a functional SNP [16], [17]. The C to G variation at IL6 rs1800796 has been shown to decrease transcriptional activity of the IL6 promoter, and carriers of CC genotype are high-expressors of IL6 [16], [17], [32]. Thus, we speculate that carriers of CC genotype have higher levels of IL6, leading to increased suppression of CYP3A5 expression and hepatoprotection. The current study showed that carriers of donor IL6 rs1800796 CC genotype were associated with faster recovery of liver function after transplantation, which is consistent with the fact that IL6 is a key molecule for liver regeneration and repair [33]. Suppression of CYP3A5 expression and hepatoprotection have opposite effects on tacrolimus metabolism. In the current study, carriers of donor IL6 rs1800796 CC genotype had a lower tacrolimus C/D ratios compared with non-carriers, indicating that the hepatoprotection effect of IL6 was greater than the suppression effect on CYP3A5 in liver transplant patients in the early postoperative period. The ability of donor IL6 rs1800796 to predict tacrolimus metabolism was less than CYP3A5 rs776746. The reason for this observation may be the opposing effects on tacrolimus metabolism of IL6 which could suppress CYP3A5 expression or provide hepatoprotection.

RETRACTED

The current study demonstrated that donor IL6 gene polymorphisms were associated with tacrolimus metabolism, not the recipient. Donor IL10 gene polymorphisms have been reported to be associated with tacrolimus metabolism [8]. Expression of IFNG and IL10 has been found to be up regulated in hepatocytes from allograft tissue after orthotopic liver transplantation [34]. There is evidence that hepatocytes can express IL6 in the HBV-infected liver microenvironment [35]. The liver has the unique capacity to regulate its growth and mass after liver injury [36]. The current data are consistent with the concept that hepatocyte secretion of IL6 may facilitate liver repair and protection after transplantation. Li et al [27] have found that serum IL18 levels were associated with tacrolimus C/D ratios and that recipient IL18 gene polymorphisms were not associated with tacrolimus C/D ratios and serum IL18 levels. We suspect that donor IL18 gene polymorphisms may be associated with tacrolimus metabolism as has been shown for IL6 in the current study.

At present, genotyping of CYP3A5 rs776746 polymorphisms has been used in clinical applications, however, it could not predict tacrolimus metabolism accurately. Our study showed that genotyping of donor IL6 rs1800796 polymorphisms could assist CYP3A5 rs776746 to predict tacrolimus metabolism more effectively. Various populations in other regions of the world may differ in certain features of genetic architecture. Whether IL6 rs1800796 is applicable to other populations with regards to tacrolimus metabolism requires further investigation. The gene-drug observations in the current study suggest that genetic factors may also affect liver transplant patient outcomes including graft and recipient survival rates. Proof of such associations requires further study.

RETRACTED

## Conclusions

Donor gene polymorphisms of IL6 play a more important role than those of recipient. Combined polymorphisms of donor CYPA5 rs776746, IL6 rs1800796, and recipient CYP3A5 rs776746 have a greater effect on tacrolimus metabolism than CYP3A5 rs776746 alone. IL6 levels may lead to individual differences in tacrolimus metabolism mainly by affecting liver function.

## References

[1] BowmanLJ, BrennanDC (2008) The role of tacrolimus in renal transplantation. Expert Opin Pharmacother 9: 635–643.1831216410.1517/14656566.9.4.635

[2] StaatzCE, TettSE (2004) Clinical pharmacokinetics and pharmacodynamics of tacrolimus in solid organ transplantation. Clin Pharmacokinet 43: 623–653.1524449510.2165/00003088-200443100-00001

[3] YuX, XieH, WeiB, ZhangM, WangW, et al (2011) Association of MDR1 gene SNPs and haplotypes with the tacrolimus dose requirements in Han Chinese liver transplant recipients. PLoS One 6: e25933.2211058210.1371/journal.pone.0025933PMC3215699

[4] Wei-linW, JingJ, Shu-senZ, Li-huaW, Ting-boL, et al (2006) Tacrolimus dose requirement in relation to donor and recipient ABCB1 and CYP3A5 gene polymorphisms in Chinese liver transplant patients. Liver Transpl 12: 775–780.1662870110.1002/lt.20709

[5] WangL, McLeodHL, WeinshilboumRM (2011) Genomics and drug response. N Engl J Med 364: 1144–1153.2142877010.1056/NEJMra1010600PMC3184612

[6] MegaJL, CloseSL, WiviottSD, ShenL, HockettRD, et al (2009) Cytochrome p-450 polymorphisms and response to clopidogrel. N Engl J Med 360: 354–362.1910608410.1056/NEJMoa0809171

[7] KleinTE, AltmanRB, ErikssonN, GageBF, KimmelSE, et al (2009) Estimation of the warfarin dose with clinical and pharmacogenetic data. N Engl J Med 360: 753–764.1922861810.1056/NEJMoa0809329PMC2722908

[8] ZhangX, WangZ, FanJ, LiuG, PengZ (2011) Impact of interleukin-10 gene polymorphisms on tacrolimus dosing requirements in Chinese liver transplant patients during the early posttransplantation period. Eur J Clin Pharmacol 67: 803–813.2135953610.1007/s00228-011-0993-8

[9] JacobsonPA, OettingWS, BrearleyAM, LeducR, GuanW, et al (2011) Novel polymorphisms associated with tacrolimus trough concentrations: results from a multicenter kidney transplant consortium. Transplantation 91: 300–308.2120642410.1097/TP.0b013e318200e991PMC3579501

RETRACTED

[10] TangHL, XieHG, YaoY, HuYF (2011) Lower tacrolimus daily dose requirements and acute rejection rates in the CYP3A5 nonexpressers than expressers. Pharmacogenet Genomics 21: 713–720.2188601610.1097/FPC.0b013e32834a48ca

[11] UesugiM, MasudaS, KatsuraT, OikeF, TakadaY, et al (2006) Effect of intestinal CYP3A5 on postoperative tacrolimus trough levels in living-donor liver transplant recipients. Pharmacogenet Genomics 16: 119–127.1642482410.1097/01.fpc.0000184953.31324.e4

[12] BirdwellKA, GradyB, ChoiL, XuH, BianA, et al (2012) The use of a DNA biobank linked to electronic medical records to characterize pharmacogenomic predictors of tacrolimus dose requirement in kidney transplant recipients. Pharmacogenet Genomics 22: 32–42.2210823710.1097/FPC.0b013e32834e1641PMC3237759

[13] de JongeH, MetalidisC, NaesensM, LambrechtsD, KuypersDR (2011) The P450 oxidoreductase *28 SNP is associated with low initial tacrolimus exposure and increased dose requirements in CYP3A5-expressing renal recipients. Pharmacogenomics 12: 1281–1291.2177072510.2217/pgs.11.77

[14] DickmannLJ, PatelSK, RockDA, WienkersLC, SlatterJG (2011) Effects of interleukin-6 (IL-6) and an anti-IL-6 monoclonal antibody on drug-metabolizing enzymes in human hepatocyte culture. Drug Metab Dispos 39: 1415–1422.2155550710.1124/dmd.111.038679

[15] TaubR (2004) Liver regeneration: from myth to mechanism. Nat Rev Mol Cell Biol 5: 836–847.1545966410.1038/nrm1489

[16] ZhangG, ZhouB, WangW, ZhangM, ZhaoY, et al (2012) A functional single-nucleotide polymorphism in the promoter of the gene encoding interleukin 6 is associated with susceptibility to tuberculosis. J Infect Dis 205: 1697–1704.2245727710.1093/infdis/jis266PMC3415858

[17] OkadaR, WakaiK, NaitoM, MoritaE, KawaiS, et al (2012) Pro-/anti-inflammatory cytokine gene polymorphisms and chronic kidney disease: a cross-sectional study. BMC Nephrol 13: 2.2223021510.1186/1471-2369-13-2PMC3297507

[18] Gabriel S, Ziaugra L, Tabbaa D (2009) SNP genotyping using the Sequenom MassARRAY iPLEX platform. Curr Protoc Hum Genet Chapter 2: Unit 2 12.10.1002/0471142905.hg0212s6019170031

[19] MacPheeIA (2012) Pharmacogenetic biomarkers: cytochrome P450 3A5. Clin Chim Acta 413: 1312–1317.2203751110.1016/j.cca.2011.10.013

[20] DalyAK (2006) Significance of the minor cytochrome P450 3A isoforms. Clin Pharmacokinet 45: 13–31.1643030910.2165/00003088-200645010-00002

[21] GervasiniG, GarciaM, MaciasRM, CuberoJJ, CaravacaF, et al (2012) Impact of genetic polymorphisms on tacrolimus pharmacokinetics and the clinical outcome of renal transplantation. Transpl Int 25: 471–480.2236969410.1111/j.1432-2277.2012.01446.x

RETRACTED

[22] ChoJH, YoonYD, ParkJY, SongEJ, ChoiJY, et al (2012) Impact of cytochrome P450 3A and ATP-binding cassette subfamily B member 1 polymorphisms on tacrolimus dose-adjusted trough concentrations among Korean renal transplant recipients. Transplant Proc 44: 109–114.2231059110.1016/j.transproceed.2011.11.004

[23] ElensL, BouamarR, HesselinkDA, HaufroidV, van der HeidenIP, et al (2011) A new functional CYP3A4 intron 6 polymorphism significantly affects tacrolimus pharmacokinetics in kidney transplant recipients. Clin Chem 57: 1574–1583.2190377410.1373/clinchem.2011.165613

[24] LownKS, KolarsJC, ThummelKE, BarnettJL, KunzeKL, et al (1994) Interpatient heterogeneity in expression of CYP3A4 and CYP3A5 in small bowel. Lack of prediction by the erythromycin breath test. Drug Metab Dispos 22: 947–955.7895614

[25] ZidekZ, AnzenbacherP, KmonickovaE (2009) Current status and challenges of cytokine pharmacology. Br J Pharmacol 157: 342–361.1937134210.1111/j.1476-5381.2009.00206.xPMC2707982

[26] LiD, ZhuJY, GaoJ, WangX, LouYQ, et al (2007) Polymorphisms of tumor necrosis factor-alpha, interleukin-10, cytochrome P450 3A5 and ABCB1 in Chinese liver transplant patients treated with immunosuppressant tacrolimus. Clin Chim Acta 383: 133–139.1756857510.1016/j.cca.2007.05.008

[27] LiY, ZouY, CaiB, YangB, YingB, et al (2012) The associations of IL-18 serum levels and promoter polymorphism with tacrolimus pharmacokinetics and hepatic allograft dysfunction in Chinese liver transplantation recipients. Gene 491: 251–255.2200866510.1016/j.gene.2011.10.008

[28] PrandotaJ (2005) Important role of proinflammatory cytokines/other endogenous substances in drug-induced hepatotoxicity: depression of drug metabolism during infections/inflammation states, and genetic polymorphisms of drug-metabolizing enzymes/cytokines may markedly contribute to this pathology. Am J Ther 12: 254–261.15891270

[29] LiuF, LiB, WangWT, WeiYG, YanLN, et al (2012) Interleukin-10-1082G/A polymorphism and acute liver graft rejection: a meta-analysis. World J Gastroenterol 18: 847–854.2237164610.3748/wjg.v18.i8.847PMC3286149

[30] AwadMR, El-GamelA, HasletonP, TurnerDM, SinnottPJ, et al (1998) Genotypic variation in the transforming growth factor-beta1 gene: association with transforming growth factor-beta1 production, fibrotic lung disease, and graft fibrosis after lung transplantation. Transplantation 66: 1014–1020.980848510.1097/00007890-199810270-00009

[31] TurnerDM, WilliamsDM, SankaranD, LazarusM, SinnottPJ, et al (1997) An investigation of polymorphism in the interleukin-10 gene promoter. Eur J Immunogenet 24: 1–8.10.1111/j.1365-2370.1997.tb00001.x9043871

RETRACTED

[32] KomatsuY, TaiH, GaliciaJC, ShimadaY, EndoM, et al (2005) Interleukin-6 (IL-6)—373 A9T11 allele is associated with reduced susceptibility to chronic periodontitis in Japanese subjects and decreased serum IL-6 level. Tissue Antigens 65: 110–114.1566374910.1111/j.1399-0039.2005.00347.x

[33] KarpSJ (2009) Clinical implications of advances in the basic science of liver repair and regeneration. Am J Transplant 9: 1973–1980.1956333410.1111/j.1600-6143.2009.02731.x

[34] Alfrey EJ, Most D, Wang X, Lee LK, Holm B, et al.. (1995) Interferon-gamma and interleukin-10 messenger RNA are up-regulated after orthotopic liver transplantation in tolerant rats: evidence for cytokine-mediated immune dysregulation. Surgery 118: 399–404; discussion 404–395.10.1016/s0039-6060(05)80351-47638757

[35] XiangWQ, FengWF, KeW, SunZ, ChenZ, et al (2011) Hepatitis B virus X protein stimulates IL-6 expression in hepatocytes via a MyD88-dependent pathway. J Hepatol 54: 26–33.2093753910.1016/j.jhep.2010.08.006

[36] FaustoN, CampbellJS (2003) The role of hepatocytes and oval cells in liver regeneration and repopulation. Mech Dev 120: 117–130.1249030210.1016/s0925-4773(02)00338-6

